# Nutritional and Biochemical Parameters Among Multiple Sclerosis Patients: A Case-Control Study

This article has been retracted.

**DOI:** 10.7759/cureus.15108

**Published:** 2021-05-19

**Authors:** Asjad Salman, Sabeeh Islam, Muhammad Awais Saleh, Khurram Khaliq Bhinder, Zainab Malik, Iqra Tahir, Muhammad A Naveed

**Affiliations:** 1 Internal Medicine, Punjab Rangers Teaching Hospital, Lahore, PAK; 2 Internal Medicine, St. Vincent Health Center, Buffalo, USA; 3 Internal Medicine, Government Khawaja Muhammad Safdar Medical College and Allied Institutions, Sialkot, PAK; 4 Radiology, Shifa International Hospital Islamabad, Islamabad, PAK; 5 Internal Medicine, Lahore General Hospital, Lahore, PAK; 6 Cardiology, Allama Iqbal Memorial Teaching Hospital, Sialkot, PAK; 7 Cardiology, Government Khawaja Muhammad Safdar Medical College and Allied Institutions, Sialkot, PAK

**Keywords:** multiple sclerosis, 25-dihydroxycholecalciferol, nutritional status, biochemical parameters, decision tree

## Abstract

Background

The pathogenesis and prognosis of multiple sclerosis (MS) is an area of active medical research. Dietary and biochemical parameters such as serum 25-dihydroxycholecalciferol, magnesium, and potassium play a role in disease progression. This study aimed to compare the nutritional status and biochemical profile of patients with and without MS.

Methodology

This case-control study included a total of 112 participants (56 in the control group and 56 in the MS group). The participants’ socioeconomic and demographic profiles, nutritional status, and biochemical details were all gathered using history, patient files, and records. The effect of these parameters on the presence of MS was evaluated using a decision tree model. Student’s t-test and Mann-Whitney U test were performed to compare these parameters.

Results

A decision tree model was developed with an accuracy rate of 86.52%. The vitamin and mineral intake of the groups showed significant statistical differences (p = 0.001). The differences were important in terms of biochemical parameters, especially serum levels of 25-dihydroxycholecalciferol and potassium.

Conclusions

The key parameters that varied between MS patients and the control group, according to the constructed decision tree, were serum levels of 25-dihydroxycholecalciferol, magnesium, calcium, potassium, and carbohydrate intake. Nutritional measures against MS can be taken based on the decision tree.

## Introduction

Multiple sclerosis (MS) is a steadily progressing disorder of the central nervous system marked by demyelinating brain and spinal cord regions [1]. The exact etiology of MS is unknown; however, genetic factors, immune system defects, and environmental factors might contribute to its etiology. Literature shows that environmental factors that influence this neurological disorder include obesity, demographics, and dietary components [1,2]. Due to the presence of epidemiological findings, some studies also hypothesize that the rise in the incidence of MS in various patient cohorts might be due to high saturated fat consumption or low intake of vitamin D [3-5]. Moreover, smoking has been proven to be a major etiological factor that contributes to the development and progression of the disease [4].

There is no proven cure for MS as there is much to be researched regarding the disease etiology, pathogenesis, and treatment. Multiple therapies including immunomodulators and steroids have been proven to ameliorate the attack episodes and to enhance the quality of life among patients suffering from MS [5]. A study reported that changes in levels of serum 25-dihydroxycholecalciferol are significantly associated with inflammatory changes, especially in diseases like MS, and such patients have lower 25-dihydroxycholecalciferol levels [5]. On the contrary, normal or elevated levels of 25-dihydroxycholecalciferol have been shown to protect patients from developing MS [5,6]. Similarly, calcium is a mineral that is essential for nerve conduction control, cell membrane stabilization, and aids in nerve impulses communication which can slow the onset or even prevent the disease [6]. Even though these studies advocate the role of these substances in disease progression, their association with other biochemical parameters such as magnesium, potassium, and nutritional parameters such as carbohydrate intake levels is understudied and needs to be evaluated. Concurrently, the existence of MS is thought to vary depending on the individual’s nutritional status and biochemical parameters. Therefore, this study aimed to assess such connections for evaluation, along with variation of these parameters in MS patients so that dietary precautions to slow the disease progression could be taken. The results of this study might help to build a causal relationship between the disease prognosis and the aforementioned factors.

## Materials and methods

This descriptive case-control study was conducted at the Government Khawaja Muhammad Safdar Medical College and Allied Institutions, Sialkot, Pakistan from January 2019 to January 2020. In terms of nutritional status and biochemical data, two groups of patients were compared. The cases included patients who had the outcome of interest, i.e., MS and those without MS. The participants’ socioeconomic status and demographic profiles, as well as their nutritional status, were determined based on the responses obtained from surveys conducted during face-to-face interviews. The biochemical information was collected from the participants’ blood samples.

The study included patients who were willing to participate, aged between 18 and 65 years, having no illness other than MS, and did not alter their eating patterns after being diagnosed with MS. A total of 196 patients met the above-mentioned inclusion criteria. To ensure the validity of biochemical analyses, patients who had not taken any disease-modifying medications, mineral supplementation, and corticosteroids in the last three months were included. The total number of patients who met these criteria was 56 (42 females and 14 males). A list of patient names who applied to the hospital’s internal medicine or endocrinology outpatient clinics during the study period was compiled to form the control group. Individuals aged between 18 and 65 years who did not have any chronic health conditions were identified and asked to participate in the current study as volunteers. To conduct sex-adjusted analyses, an equal number of male and female (42 females and 14 males) participants were selected as controls.

Participants’ general characteristics, health status, and eating habits were studied. Participants were asked to share their average daily intake of the most commonly consumed nutrients through a well-organized survey. The program Ebispro for Windows was used to test the average 24-hour retrospective food intake records of the study participants. The participants’ energy and nutrient intake were measured. A total of 33 food and beverage-related questions were used to collect data on daily average food intake. Participants were asked how often they would eat those foods and beverages daily. The total daily energy intake, as well as macro and micronutrient intake, were calculated based on the responses.

For the summer and winter seasons, the reference values for 25-dihydroxycholecalciferol were set at 20-120 ng/mL and 10-60 ng/mL, respectively, based on the hospital’s laboratory requirements. The Beckman Coulter AU-5800 (Beckman Coulter, Brea, CA) unit was used to calculate all parameters except serum 25-dihydroxycholecalciferol. The level of 25-dihydroxycholecalciferol in the blood was measured using the chemiluminescence immunoassay method on a Beckman Coulter Dlx-800. The spectrophotometry method was used to evaluate serum Ca, Mg, and inorganic phosphate levels, while the ion-selective electrode method was used to determine serum K levels. Spectrophotometric methods were used to quantify lipid profile values. The serum levels of alanine aminotransferase, aspartate aminotransferase, and alkaline phosphatase were measured using a kinetic spectrophotometric tool, while immunoturbidimetric methods were used to measure inflammatory markers like C-reactive protein.

Shapiro-Wilk normality tests were used to assess the normality of the data. The Chi-square test was used to evaluate whether there was a relationship between the variables. The variations between MS patients and healthy people in terms of socioeconomic and demographic factors, nutritional status, and biochemical information were demonstrated using a decision tree model. The statistical significance standard for all tests was set at 0.05. Rapid Miner Studio version 8.2 was used to build the decision tree model. SPSS Statistics for Windows, version 25.0 (IBM Corp., Armonk, NY) was used to perform all statistical calculations.

## Results

The frequency analysis showing the socioeconomic and demographic characteristics of the participants is shown in Table 1.

**Table 1:** Socioeconomic and demographic characteristics of the study population. MS: multiple sclerosis

Parameter		Control group (n = 56)	MS group (n = 56)	Total (N = 112)
Gender	Male	42 (75%)	42 (75%)	84 (75%)
	Female	14 (25%)	14 (25%)	28 (25%0
Age	18-30 years	17 (30.4%)	14 (25%)	31 (27.7%)
	31-50 years	32 (57.1%)	35 (62.5%)	67 (59.8%)
	Above 51 years	7 (12.5%)	7 (12.5%)	14 (12.5%)
Education	Below high school	11 (19.6%)	32 (57.1%)	43 (38.4%)
	High school	14 (25%)	15 (26.8%)	29 (25.9%)
	University	31 (55.4%)	9 (16.1%)	40 (35.7%)
Marital status	Married	40 (71.4%)	46 (82.1%)	86 (76.8%)
	Unmarried	16 (28.6%)	10 (17.9%)	26 (23.2%)
Place of living	Urban	55 (98.21%)	47 (83.92%)	102 (91.1)
	Rural	1 (1.8%)	9 (16.1%)	10 (8.9%)

The average daily energy, macronutrient, and micronutrient intake of the control and MS groups were compared to see whether there were statistically significant differences. In this study, descriptive statistics, as well as comparisons of participants’ nutritional status, were presented. Between the control and MS groups, there were no statistically significant differences in percentage lipid, carbohydrate, protein, cholesterol, calcium, phosphorus, vitamin B2, vitamin B12, and zinc intake (P values were 0.383, 0.694, 0.219, 0.132, 0.119, 0.056, 0.123, 0.650, and 0.548, respectively). However, there were significant statistical variations between the control and MS groups’ measured carbohydrate, lipid, potassium, vitamin B1, and B6 intake. In general, the control group had higher energy and nutrient intake than the MS group.

Participants’ biochemical data were collected to look at the potential discrepancies between the control and MS groups. Descriptive statistics, as well as references to the biochemical data of the participants, were shown. There were statistically significant differences in serum levels of calcium, magnesium, potassium, vitamin D, and low-density lipoprotein between the groups. The difference was particularly noticeable in serum levels of 25-dihydroxycholecalciferol and potassium. The serum 25-dihydroxycholecalciferol level was slightly lower (8.9 ± 4.0 ng/mL) in the MS group than the control group (18.9 ± 11.0 ng/mL). Similarly, the MS group had a slightly lower mean serum potassium level than the control group (4.11 ± 0.41 mEq/L versus 4.45 ± 0.41 mEq/L, respectively; p = 0.001).

A decision tree model was developed to compare the threshold values of certain parameters in healthy people and MS patients based on nutritional status and biochemical information obtained from the participants. The built tree was difficult to investigate as there were so many features gathered from the participants. Therefore, a forward selection approach was used to determine the best subset of features for simplifying the tree. The five characteristics that made up the decision tree that produced the best classification results were serum levels of vitamin D, magnesium, calcium, and potassium, and carbohydrate intake.

Following the arrows from the top to bottom and paying attention to the feature’s limit values helps in the interpretation of the tree. In this study, 29 participants had a serum 25-dihydroxycholecalciferol level of less than 15.40 ng/mL, a serum magnesium level of less than 2.29 mg, a serum calcium level of less than 9.56 mg/dL, and a potassium intake of less than 1,798.05 mg. The constructed tree, as a descriptive method, is ideal for comparing parameter differences between the control and MS groups. Physicians may be able to take dietary measures based on the tree’s descriptive findings. The tree is shown in Figure 1.

**Figure 1:** Decision tree hierarchy representing the relative discriminating power of the key variables. 25(OH)D: 25-dihydroxycholecalciferol; CHO: carbohydrate; MS: multiple sclerosis

The textual representation of the decision tree is shown in Figure 2.

**Figure 2:** Textual representation of the tree. Each line of text corresponds to a node or a leaf, and the indentation reflects the tree level. For a node, the split condition is displayed; for a leaf, the assigned class label is shown. 25(OH)D: 25-dihydroxycholecalciferol; CHO: carbohydrate; MS: multiple sclerosis

## Discussion

Unlike several previous studies that compared only serum 25-dihydroxycholecalciferol levels of MS patients and healthy people, the current research focused on building a decision tree model to reveal the threshold values of certain parameters in both healthy people and MS patients. This decision tree was used to assess the critical values for 25-dihydroxycholecalciferol serum levels, magnesium, calcium intake, and potassium and CHO intake. As stated in the study, MS has a wide range of clinical characteristics, topography of involvement, and natural history variations, as seen in the western and eastern hemispheres [7]. The study design has a significant drawback in terms of determining causality. Although it is impossible to conclude the causes of MS solely based on descriptive discrepancies, the decision tree’s selected parameters indicate that the related variables are the most distance between the two classes. That is, these parameters may serve as a starting point for a well-designed cohort study, allowing for a wider quest for causality. Only mean values could be compared in the current study due to a lack of research in the literature on essential value assessment for MS patients. The parameters of the built decision tree have frequently been examined as potential causes of MS, according to the literature review.

The level of serum 25-dihydroxycholecalciferol, which is thought to be a key variable, varies between healthy people and MS patients. Because 25-dihydroxycholecalciferol levels are known to vary by season, different reference values for 25-dihydroxycholecalciferol were used in this study for winter and summer seasons. The 25-dihydroxycholecalciferol levels of the control and MS groups were substantially different during both summer and winter seasons (P values of 0.029 and 0.001, respectively). Due to the nearly identical number of patients in both groups who had their measurements taken in winter (or summer), the distinction was made without regard to the season. The MS group had slightly lower levels of serum 25-dihydroxycholecalciferol (8.87 ± 4.02 ng/mL) than the control group (18.86 ± 11.04 ng/mL).

Similar results were obtained in other studies [8,9]. Deficiency in 25-dihydroxycholecalciferol has been linked to an increased risk of MS in numerous studies. Furthermore, three studies found an inverse relationship between MS prevalence and sunlight exposure, which is believed to be the primary source of vitamin D; six among veterans from the United States and Australia [10,11].

Magnesium is needed for nerve transmission as well as neuromuscular conduction. It also protects against excessive excitation, which can lead to neuronal cell death, and has been linked to various neurological disorders [12]. Magnesium is essential for axon stabilization and influences neurotransmitter release. Nerve conduction velocity increases and the threshold for axon stimulation decreases when magnesium levels are low [13]. Magnesium is a mineral that has a lot of potential for preventing and treating neurological conditions because of its essential role within the nervous system [14]. Consequently, differences in serum magnesium levels between the control and MS groups seem rational. Indeed, serum magnesium levels in the MS group (1.97 ± 0.18 mg/dL) were found to be slightly lower than those in the control group (2.43 ± 2.82 mg/dL, P = 0.037) in the current study. The majority of previous studies support these findings [15].

The serum calcium levels (9.14 ± 0.63 mg/dL) in the MS group were statistically significantly lower than the control group (9.33 ± 0.92 mg/dL; P = 0.004) in the current study. Similar results were found in another study [16]. There may be many explanations for this. Glucocorticoids, an anti-inflammatory hormone released by the adrenal glands, are used to treat acute exacerbation or relapses in people with MS. Because glucocorticoids reduce intestinal calcium absorption while increasing renal calcium excretion, they are used to treat osteoporosis [17], calcium deficiency may have been present in MS patients. Furthermore, when vitamin D deficiency or insufficiency occurs, intestinal calcium absorption decreases, resulting in a subtle decrease in serum calcium levels [18]. In our study, low vitamin D levels in MS patients may have resulted in a decrease in calcium absorption. In addition, increased calcium losses in women due to menopause may have influenced calcium intake.

Low-carbohydrate diets are linked to increased ambulation and physical exercise in people with MS [19]. Carbohydrate-rich diets have been linked to lipid and glucose metabolism problems in MS patients [20]. MS patients consumed substantially less carbohydrate than healthy individuals in the current study (P = 0.001). Because of their physical activity limitations, it is believed that MS patients consume a balanced diet and restrict their carbohydrate intake or consume fast food. This situation may seem to be more of an obligation than a deliberate choice [21]. According to our results, MS patients are determined to eat more fat and protein while consuming less carbohydrate than the general population. Moreover, some studies compared male and female MS patients in terms of their carbohydrate intake [22].

By analyzing nutritional status and biochemical parameters of people with and without MS, the observations and findings of this study aimed to contribute to the literature in terms of MS recognition. A new research field was attempted to be developed on the determination of critical values for MS patients by providing a decision tree model. The constructed tree, as a descriptive method, is ideal for comparing parameter differences between the control and MS classes. The key parameters that vary between an MS patient and a healthy individual are serum levels of vitamin D, magnesium, calcium, potassium intake, and carbohydrate intake, according to the report. It is important to remember that the parameters used to construct the decision tree are not the cause of MS. The aim of this study was not to find a connection between the two events.

Having a retrospective outlook and a single-centered study design account for a few limitations in our study. Further multicentric cohort studies will help to develop the casual association between the disease and nutritional parameters. However, the results of our study open up new questions regarding the relationship of nutritional and biochemical parameters with MS.

## Conclusions

The key parameters that varied between an MS patient and a healthy individual, according to the constructed decision tree, were serum levels of 25-dihydroxycholecalciferol, magnesium, calcium, and potassium, and carbohydrate intake. Nutritional measures against MS can be taken based on the results of this study. The discrepancies between MS patients and healthy individuals should be identified in terms of certain parameters in prospective cohort studies. The findings show that vitamin D, magnesium, and calcium levels in the blood are predicted to be lower in MS patients.
